# Modulation of Mitochondrial Quality Control Processes by BGP-15 in Oxidative Stress Scenarios: From Cell Culture to Heart Failure

This article has been retracted.

**DOI:** 10.1155/2021/6643871

**Published:** 2021-02-27

**Authors:** Orsolya Horvath, Katalin Ordog, Kitti Bruszt, Nikoletta Kalman, Dominika Kovacs, Balazs Radnai, Ferenc Gallyas, Kalman Toth, Robert Halmosi, Laszlo Deres

**Affiliations:** ^1^1st Department of Medicine, University of Pecs, Medical School, Pecs, Hungary; ^2^Szentágothai Research Centre, University of Pecs, Pecs, Hungary; ^3^Department of Biochemistry and Medical Chemistry, University of Pecs, Medical School, Pecs, Hungary; ^4^HAS-UP Nuclear-Mitochondrial Interactions Research Group, 1245 Budapest, Hungary

## Abstract

Heart failure (HF) is a complex chronic clinical disease characterized by among others the damage of the mitochondrial network. The disruption of the mitochondrial quality control and the imbalance in fusion-fission processes lead to a lack of energy supply and, finally, to cell death. BGP-15 (O-[3-piperidino-2-hydroxy-1-propyl]-nicotinic acid amidoxime dihydrochloride) is an insulin sensitizer molecule and has a cytoprotective effect in a wide variety of experimental models. In our recent work, we aimed to clarify the mitochondrial protective effects of BGP-15 in a hypertension-induced heart failure model and “in vitro.” Spontaneously hypertensive rats (SHRs) received BGP-15 or placebo for 18 weeks. BGP-15 treatment preserved the normal mitochondrial ultrastructure and enhanced the mitochondrial fusion. Neonatal rat cardiomyocytes (NRCMs) were stressed by hydrogen-peroxide. BGP-15 treatment inhibited the mitochondrial fission processes, promoted mitochondrial fusion, maintained the integrity of the mitochondrial genome, and moreover enhanced the de novo biogenesis of the mitochondria. As a result of these effects, BGP-15 treatment also supports the maintenance of mitochondrial function through the preservation of the mitochondrial structure during hydrogen peroxide-induced oxidative stress as well as in an “in vivo” heart failure model. It offers the possibility, which pharmacological modulation of mitochondrial quality control under oxidative stress could be a novel therapeutic approach in heart failure.

## 1. Introduction

Several studies have demonstrated that mitochondria, the powerhouse of cells are damaged in heart failure as well as in hypertension-induced cardiac remodelling [1–3]. The balance of fusion and fission processes that regulate mitochondrial dynamics is essential for maintaining energy production [4, 5]. The most important fusion proteins in the regulation of mitochondrial dynamics are the optic atrophy 1 (OPA1) and the mitofusin 1 and 2 (MFN1, MFN2) proteins, while the fission processes of mitochondria are controlled by dynamin-related protein 1 (DRP1) [6–8].

In heart failure due to the increased ROS production, fission processes become predominant, resulting in fragmented mitochondrial network, which is unable to perform its function of providing energy to the cell; thereby, mitochondrial fragmentation can induce cell death [2, 4, 9, 10]. The subject of numerous researches is the regulation of mitochondrial dynamics as a new therapeutic target in cardiovascular diseases [6, 11–14].

BGP-15 (O-[3-piperidino-2-hydroxy-1-propyl]-nicotinic acid amidoxime dihydrochloride) is an insulin sensitizer molecule and has a cytoprotective effect in a wide variety of experimental models (Figure 1). BGP-15 protects against oxidative stress [15–17], promotes mitochondrial fusion [18], inhibits the mitogen-activated protein kinase (MAPK) activation [19–22], and improves cardiac function [21–23], but its specific intracellular target is still unknown.

This study was aimed to further characterize the mitochondrial effects of BGP-15 in a chronic hypertension-induced heart failure animal model and “in vitro” using primer neonatal rat cardiomyocytes (NRCM). We studied the effect of BGP-15 on the processes of mitochondrial quality control, particularly on fusion-fission processes, on mitochondrial biogenesis as well as on mitochondrial function.

## 2. Materials and Methods

### 2.1. Ethics Statement

Animals received care according to the Guide for the Care and Use of Laboratory Animals published by the US National Institute of Health and the experiment was approved by the Animal Research Review Committee of the University of Pecs, Medical School (Permit number: BA02/2000-54/2017).

### 2.2. Animal Model

15-month-old male Wistar Kyoto (WKY) and spontaneously hypertensive rats (SHR) (Charles River Laboratories, Budapest, Hungary) were used. Two animals were housed per cage under standardized conditions throughout the experiment, with 12 hours of dark-light cycle in solid-bottomed polypropylene cages and received commercial rat chew and water ad libitum. 8 of the 24 animals were sacrificed at the beginning of the experiment, as a baseline (SHR-Baseline). The surviving 16 SHRs were randomly divided into two groups: SHR-B and SHR-C. SHR-B group was treated with the water-soluble BGP-15 (25 mg/b.w. in kg/day, *n* = 8), while SHR-C group received only placebo (*n* = 8, SHR-C) per os for 18 weeks. BGP-15 was a gift from N-Gene Inc. (New York, NY, USA). The dosage of BGP-15 administered in the drinking water was based on preliminary data about the volume of daily water consumption. WKY rats were used as age-matched controls (*n* = 8). At the end of the 18-week long treatment period, animals were sacrificed, and blood was collected to determine the concentration of plasma brain-derived natriuretic peptide (BNP). Hearts were removed, atria and great vessels were trimmed from the ventricles, and the weight of the ventricles was measured; then, it was normalized to the body mass and to the length of the right tibia (indices of cardiac hypertrophy). Hearts were fixed in modified Kranovsky fixative for transmission electron microscopy or freeze-clamped for Western blot analysis. The levels of proteins which are involved in the processes of mitochondrial dynamics and biogenesis were monitored by Western blot analysis. In our research, the following group notations were used according to the applied treatment: WKY: age-matched normotensive Wistar Kyoto rats; SHR-Baseline: 15-month-old spontaneously hypertensive rats; SHR-C: 19-month-old spontaneously hypertensive rats received placebo for 18 weeks; SHR-B: 19-month-old spontaneously hypertensive rats received BGP-15 for 18 weeks.

### 2.3. Neonatal Rat Cardiomyocyte (NRCM) Cell Culture

Cardiomyocytes were isolated using the Pierce™ Primary Cardiomyocyte Isolation Kit (Life Technologies, Carlsbad, CA, USA #88281) from 1-3-day-old neonatal Wistar rats. The animals were sacrificed, and then, their hearts were removed and minced into 1-3 mm^3^ pieces. The pieces were digested with an enzyme complex (Cardiomyocyte Isolation Enzyme 1 (with papain) and Cardiomyocyte Isolation Enzyme 2 (with thermolysin)). After the tissue became primarily a single-cell suspension, the cells had been plated in 6-well plates with a density of 2.5 × 10^6^ cell/well with specific Dulbecco's Modified Eagle Medium (DMEM) for Primary Cell Isolation containing 10% fetal bovine serum (FBS), 100 IU/mL penicillin and 100 *μ*g/mL streptomycin. The medium was replaced 24 hours later with fresh Complete DMEM for Primary Cell Isolation containing Cardiomyocyte Growth Supplement, which inhibited the division of fibroblasts and therefore maintained the cardiomyocyte suspension in high purity during the culture period. NRCMs were cultivated in normal culture conditions, 37°C, saturated humidity atmosphere of 95% air and 5% CO2. Fresh medium was added every 2-3 days.

### 2.4. Treatments of Neonatal Rat Cardiomyocytes

On the day of the experiments, cells were washed once in PBS and added fresh medium and, then, treated with 150 *μ*M H_2_O_2_ with or without 50 *μ*M BGP-15 for 0.5 hours. The following groups were created according to the applied treatment: Control group: cells without any treatment; BGP-15 group: cells with only 50 *μ*M BGP-15 for 0.5 hours; H_2_O_2_ group: cells with 150 *μ*M H_2_O_2_ for 0.5 hours; H_2_O_2_+BGP-15 group: cells with 150 *μ*M H_2_O_2_ and 50 *μ*M BGP-15 for 0.5 hours.

### 2.5. Determination of Plasma B-Type Natriuretic Peptide Level

Blood samples were collected into Vacutainer tubes containing EDTA and aprotinin (0.6 IU/ml) and centrifuged at 1600 g for 15 minutes at 4°C to separate plasma, which was collected and kept at −70°C. Plasma B-type natriuretic peptide-32 levels (BNP-32) were determined by Enzyme-Linked Immunosorbent Assay method (BNP-32, Rat BNP 32 ELISA Kit, Abcam, ab108815CA, USA) as the datasheet recommends.

### 2.6. Transmission Electron Microscopy

For electron microscopy analysis, hearts were perfused retrogradely through the aortic root with ice-cold PBS to wash out the blood and then with modified Kranovsky fixative (2% paraformaldehyde, 2.5% glutaraldehyde, 0.1 M Na-cacodylate buffer, pH 7.4, and 3 mM CaCl_2_). 1 mm thick sections were cut from the free wall of the left ventricle. Dehydrated blocks were embedded in Durcupan resin. From the embedded blocks, semithin sections of 500 nm and ultrathin sections of 50 nm were cut with a Leica ultramicrotome and mounted either on mesh or on Collodion-coated (Parlodion, Electron Microscopy Sciences, Fort Washington, PA) single-slot, copper grids. Additional contrast was provided to these sections with uranyl acetate and lead citrate solutions, and the preparations were examined with a JEOL 1200EX-II electron microscope. 4 animals from each group, 3–5 blocks from each animal were used. The area of the interfibrillar mitochondria (IFM) was measured by freehand polygon selection (n~500/group) using the ImageJ software.

### 2.7. Western-Blot Analysis

#### 2.7.1. Total Western Blot Sample Preparation from Cardiac Tissue

50 milligrams of heart samples were homogenized in ice-cold Tris buffer (50 mmol/l, pH 8.0) containing protease inhibitor (1 : 100; Sigma-Aldrich Co., #P8340) and phosphatase inhibitor (1 : 100; Sigma-Aldrich Co., #P5726) and 50 mM sodium vanadate. The supernatants were harvested in 2x concentrated sodium dodecyl sulfate- (SDS-) polyacrylamide gel electrophoresis sample buffer.

#### 2.7.2. Fractionated Western Blot Sample Preparation from Cardiac Tissue

100 milligrams of heart tissues were minced in ice-cold isolation solution (150 mM NaCl, 50 mM TRIS, and 1 mM EDTA), protease inhibitor (1 : 100; Sigma-Aldrich Co., #P8340), and phosphatase inhibitor (1 : 100; Sigma-Aldrich Co., #P5726)). Samples were disrupted on ice with gently Turrax and, then, processed in a Potter-Elvehjem tissue homogenizer. Samples were centrifuged for 12 minutes at 750 g. Supernatants containing the cytosolic and mitochondrial fractions were aspirated and the precipitated nuclear fractions were harvested in 2x SDS–polyacrylamide gel electrophoresis sample buffer and denatured at 95°C for 5 minutes. Supernatants were then centrifuged for 12 minutes at 11.000 g to gain cytosolic fraction in the supernatant and mitochondrial fraction in the precipitate. Samples were harvested separately in 2x SDS–polyacrylamide gel electrophoresis sample buffer and denatured at 95°C for 5 minutes.

#### 2.7.3. Total Western-Blot Sample Preparation from NRCM Cell Culture

After the appropriate treatment, cells were harvested. The cell pellet was suspended in ice-cold PBS buffer and, then, centrifuged for 5 min at 1,200 rpm at room temperature. The pellets were suspended in 300 *μ*L NP-40 lysis buffer (Amresco, J619) containing protease inhibitor (1 : 100; Sigma-Aldrich Co., #P8340) and phosphatase inhibitor (1 : 100; Sigma-Aldrich Co., #P5726). The samples were shaken for 30 min at 4°C; then, they were centrifuged for 20 min (4°C 12,000 rpm). 4x concentrated SDS-polyacrylamide gel electrophoresis sample buffer was added to each sample.

#### 2.7.4. Fractionated Western Blot Sample Preparation from NRCM Cell Culture

The cell pellet was suspended in an ice-cold isolation solution (0.5 mM TRIS, 1 M EGTA, and 0.4 M sucrose) containing 0.5 mM sodium metavanadate, 0.05 M EDTA, and protease inhibitor (1 : 100; Sigma-Aldrich Co., #P8340). Samples were disrupted on ice by Turrax and, then, processed by a Potter-Elvehjem tissue homogenizer. Centrifugation was carried out for 15 minutes at 750 g. The nuclear fraction in the precipitate was harvested in 72% trichloroacetic acid. Subsequently, supernatants were aspirated and centrifuged for 15 minutes at 10.000 g to gain cytosolic fraction in the supernatant and mitochondrial in the precipitate. Samples were harvested separately in 72% trichloroacetic acid. The precipitated fractions were centrifuged for 10 minutes at 15.000 g. Each precipitate was harvested separately in a 50 mM TRIS and SDS-polyacrylamide gel electrophoresis sample buffer. The samples were shaken for overnight at 4°C and denatured at 95°C for 5 minutes. After that, they were centrifuged for 10 minutes at 15.000 g, and the supernatants were collected as the mitochondrial fraction.

#### 2.7.5. Electrophoresis and Transfer of Proteins

After the preparation, the tissue and cell culture samples were processed in the same manner. Protein levels were measured with Nanodrop. Glyceraldehyde 3-phosphate dehydrogenase (GAPDH; 1 : 1000; Cell Signaling #2118) and pyruvate dehydrogenase (PDC; 1 : 1000; Cell Signaling #3205) were used as a representative loading control. Proteins were separated on 12% SDS-polyacrylamide gel and transferred to nitrocellulose membranes. After blocking (2 h with 5% BSA in Tris-buffered saline contained with 1% Tween-20), membranes were probed overnight at 4°C with primary antibodies recognizing the following antigens: optic atrophy 1 (OPA1; 1 : 1000; Cell Signaling #80471), mitofusin-1 (MFN1; 1 : 1000; Abcam ab57602), mitofusin-2 (MFN2; 1 : 1000; Cell Signaling #9482), dynamin-related protein 1 (DRP1; 1 : 1000; Cell Signaling #8570), phosphor-specific DRP1 Ser637 (1 : 500; Cell Signaling #4867), phosphor-specific DRP1 Ser616 (1 : 500; Cell Signaling #3455), voltage-dependent anion channel (VDAC; 1 : 1000; Cell Signaling #4661), mitochondrial fission 1 protein (FIS1; 2 *μ*g/mL, Abcam, ab71498), peroxisome proliferator-activated receptor gamma coactivator 1-alpha (PGC-1*α*; 1 : 1000; Novus Biologicals, NBP1-04676), cAMP response element-binding protein (CREB; 1 : 1000; Cell Signaling #4820), phosphor-specific cAMP response element-binding protein Ser133 (1 : 1000; Cell Signaling #9198), anti-NADH dehydrogenase Fe-S protein 1 (NDUFs1, Novus Biologicals, NBP1-31142, 1 : 1000), and anti-Ubiquinol-cytochrome c reductase core protein I (UQCRC1, Novus Biologicals, NBP2-03825, 1 : 1000). Membranes were washed six times for 5 min in Tris-buffered saline (pH 7.5) containing 0.2% Tween (TBST) before the addition of horseradish peroxidase-conjugated secondary antibody (goat anti-rabbit IgG, Sigma Aldrich Co. A0545, 1 : 3000 dilution; rabbit anti-mouse IgG, Sigma Aldrich Co., A9044, 1 : 5000 dilution). Membranes were washed six times for 5 min in TBST, and then, the antibody-antigen complexes were visualized by enhanced chemiluminescence. The results of Western blots were quantified using the NIH ImageJ program.

### 2.8. Capillary Electrophoresis Immunoassay

Due to the limited availability of primary neonatal cardiomyocytes and the lower protein concentration of the fractionated samples made from it, the more sensitive capillary immunoassay method with less sample requirements and higher throughput is more suitable for measurement. Simple western analysis (Wes) was performed on a Wes system (ProteinSimple, product number 004–600) according to the manufacturer's instructions using a 12-230 kDa Separation Module (ProteinSimple SM-W004) and either the Anti-Rabbit Detection Module (ProteinSimple DM-001) or the Anti-Mouse Detection Module (ProteinSimple DM-002), depending on the primary used antibody. Subcellular NRCM samples were mixed with Fluorescent Master Mix and heated at 95°C for 5 min. The samples, blocking reagent (antibody diluent), primary antibodies (in antibody diluent), HRP-conjugated secondary antibodies, and chemiluminescent substrate, were pipetted into the plate (part of Separation Module). Instrument default settings were used: stacking and separation at 475 V for 30 min; blocking reagent for 5 min, primary and secondary antibody both for 30 min; Luminol/peroxide chemiluminescence detection for ~15 min (exposures of 1-2-4-8-16-32-64-128-512 s). The resulting electropherograms were inspected to check whether automatic peak detection required any manual correction.

### 2.9. Evaluation of Mitochondrial Fragmentation with Fluorescent Microscopy

NRCM cells were seeded at a density of 10^5^ cells/well in 6 well plates on glass coverslips with 1% gelatin coating and cultured at least for 2 days before the experiment. On the day of the experiment, cells were washed once in PBS and added fresh medium and, then, treated with H_2_O_2_ with or without BGP-15. After the appropriate treatment, coverslips were rinsed in PBS and were added 75 nM MitoTracker Red CMXRos dissolved in serum-free DMEM and incubated for 30 min at 37°C. After the incubation, coverslips were rinsed in PBS, and the mitochondrial network was visualized by a Nikon Eclipse Ti-U fluorescent microscope equipped with a Spot RT3 camera using a 60x objective and epifluorescent illumination.

### 2.10. Quantification of Mitochondrial DNA (mtDNA) Damage by Real-Time PCR

After the appropriate treatment, cells were harvested, and total DNA was isolated using GenElute™ Mammalian Genomic DNA Miniprep Kits (Sigma-Aldrich # G1N350-1KT). Real-time DNA amplification was performed using a CFX96 Touch Real-Time PCR Detection System (Bio-Rad) as we performed earlier [25]. The following rat primer sequences were used: SRPCR (210 bp) forward: 5′-ATGCACGATAGCTAAGACCCAA-3 ′; reverse: 5 ′-CTGAATTAGCGAGAAGGGGTA-3′ and LRPCR (14958 bp) forward: 5 ′-ATTTTCTCCCAGTTACGAAAG-3 ′, reverse: 5 ′-CTTGGTAAGTAAATTTCTTTCTCC-3 ′. Short fragment, cytochrome c oxidase subunit 1 (COX1), cytochrome c oxidase subunit 3 (COX3), and *β*-actin were done using a Brilliant II QPCR Master Mix (Agilent Technologies, # 600804). The final SRPCR, COXI, COXIII, and *β*-actin cycling parameters followed hot start of 10 min at 95°C, followed by 30 sec at 95°C, 1 min at 60°C, and 30 sec at 72°C for 40 cycles. LRPCR was done using PfuUltra II Hotstart 2x Master Mix (Agilent Technologies, #600852). The final LRPCR cycling parameters followed manufacturer's recommendations: hot start of 2 min at 92°C, followed by 15 sec at 92°C, 30 sec at 50°C, and 8 : 00 min at 68°C for 40 cycles. The relative mitochondrial DNA content was determined by real-time PCR, using COX1 and COX3 primers, normalized to a nuclear-encoded *β*-actin gene. The following rat primer sequences were used: COX1 (199 bp) forward: 5 ′-CACAGTAGGGGGCCTAACAG-3 ′, reverse: 5 ′-CAAAGTGGGCTTTTGCTCAT-3 ′; COX3 (244 bp) forward 5 ′-TCAGGAGTCTCAATTACATG-3 ′, reverse: 5 ′-CGTAGTAGACAGACAATTAGG-3 ′; *β*-actin (191 bp) forward 5 ′-GCGGTGACCATAGCCCTCTTT-3 ′, reverse: 5 ′-TGCCACTCCCAAAGTAAAGGGTCA-3 ′. The software automatically generated crossing points and calculation of mtDNA damage was made using the *Δ*2^Ct^ method. EvaGreen dye was used (Biotium # 31000).

### 2.11. Mitochondrial Membrane Potential Measurement with JC-1 Assay

The mitochondrial membrane potential (*ΔΨ*m) was measured using the mitochondrial membrane potential specific fluorescent probe, JC-1 (Enzo Life Sciences, ENZ-52304) as we performed it earlier [25]. NRCM cells were seeded on glass coverslips coated with gelatin and cultured for at least 2 days before the experiment. After the treatment, cells were washed in PBS and incubated for 15 min at 37°C in media containing 5 *μ*g/mL JC-1. When excited at 488 nm, the dye emits red fluorescence (590 nm) at high *ΔΨ*m and green (530 nm) at low *ΔΨ*m. Following incubation, the cells were washed once with PBS and then imaged with a Nikon Eclipse Ti-U fluorescent microscope equipped with a Spot RT3 camera using a 60x objective and epifluorescent illumination. All experiments were repeated three times. Fluorescent signals were quantified by using the ImageJ software (NIH, Bethesda, MD, USA).

### 2.12. Evaluation of the Mitochondrial Energy Metabolism and Function

As we described earlier, Agilent Seahorse Extracellular Flux (XFp) Analyzer (Agilent Technologies, (Santa Clara, CA, USA)) was used to determine the NRCM cells' oxygen consumption rate (OCR) [25]. NRCM cells were seeded in XFp Miniplate at a density of 4 × 10^4^ cells/well in 80 *μ*L complete growth medium (DMEM for Primary Cell Isolation containing 10% FBS, 100 IU/mL penicillin and 100 *μ*g/mL streptomycin) and incubated at 37°C, 5% CO_2_ for 2 days. On the day before the experiment, sensor cartridges were hydrated in XFp calibrant and maintained at 37°C without CO_2_ overnight. On the day of the assay, after subjecting cells to the appropriate treatment, DMEM for Primary Cell Isolation medium was replaced by Agilent Seahorse XF Base Medium containing 1 mM pyruvate, 2 mM glutamine, and 10 mM glucose (adjusted pH to 7.4 with 0.1 N NaOH). Before measurement, different compounds were loaded into the appropriate ports of a hydrated sensor cartridge (10 *μ*M oligomycin, 10 *μ*M FCCP, and 5 *μ*M rotenone/antimycin). Three measurements were performed after each injection. OCR was used to determine mitochondrial energy metabolism. The parameter values, including basal respiration, maximal respiration, ATP-associated OCR, and spare respiratory capacity, were determined according to the Seahorse XFp Cell Mito Stress user guide protocol. Data were analyzed using the Seahorse XF test report analysis.

### 2.13. Analysis of Citrate Synthase Activity in NRCM Cells

NRCM cells were seeded at a density of 10^6^ cells/well in 6-well plates and cultured. After the appropriate treatment, cells were harvested; the cell pellet was suspended in ice-cold citrate synthase cell lysis buffer and, then, centrifuged for 5 min at 4°C at 10,000 x g; then, the supernatant was collected for further use. Citrate synthase was measured using a kit from Sigma Aldrich (MAK193) following the manufacturer's instruction. The absorbance was recorded at 412 nm every 5 minutes for 50 minutes. The colorimetric product (GSH) was proportional to the enzymatic activity of citrate synthase and normalized to the quantity of cells.

### 2.14. Statistical Analysis

Statistical analysis was performed by analysis of variance, and all of the data were expressed as the mean ± SEM. The homogeneity of the groups was tested by F-test (Levene's test). There were no significant differences among the groups. Comparisons among groups were made by one-way ANOVA with a post hoc correction (SPSS for Windows, version 21.0). The Student's *t*-test was used to compare the mean values of two groups. A value of *p* < 0.05 was considered statistically significant.

## 3. Results

### 3.1. In Vivo Results

#### 3.1.1. Effect of BGP-15 Administration on Gravimetric Parameters and on BNP Level

At the beginning of the study, the body weight of WKY rats was significantly higher than the SHR rats (WKY: 391.51 ± 8.64 g, SHR-C: 340.66 ± 6.74 g, SHR-B: 347.4 ± 10.38 g; *p* < 0.05, WKY vs. SHR groups; Table 1). Similar observation can be made at the end of the study (WKY: 403.22 ± 10.35 g, SHR-C: 352.13 ± 6.86 g, SHR-B: 365.29 ± 6.82 g; *p* < 0.05 WKY vs. SHR groups). At the end of the study, heart weights (HW) and ventricles weight (VW) were significantly increased in the SHR groups compared to the WKY group (HW: WKY: 1.11 ± 0.03 g, SHR-C: 1.41 ± 0.03 g, SHR-B: 1.28 ± 0.02 g; *p* < 0.01 SHR-B and SHR-C vs.WKY, *p* < 0.05 SHR-B vs. SHR-C; VW: WKY: 0.98 ± 0.03 g, SHR-C: 1.27 ± 0.02 g, SHR-B: 1.12 ± 0.02 g; *p* < 0.05 SHR-groups vs. WKY). The ratio of ventricular weight to body weight (VW/BW) was increased markedly in SHR groups compared to WKY animals (VW/BW (mg/g): WKY: 2.43 ± 0.07, SHR-C: 3.60 ± 0.04, SHR-B: 3.07 ± 0.09; *p* < 0.01 SHR groups vs. WKY, *p* < 0.05 SHR-B vs. SHR-C). Ventricular weight to the length of right tibia ratio (VW/TL) was also significantly increased (VW/TL (mg/mm): WKY: 21.43 ± 0.71, SHR-C: 29.14 ± 0.14, SHR-B: 24.81 ± 0.53; *p* < 0.05 SHR-groups vs. WKY). BGP-15 treatment caused a significant moderation of these ratios (*p* < 0.05 SHR-B vs. SHR-C).

By the end of the treatment, the plasma BNP level increased significantly in the SHR-C group compared to the WKY group (BNP (pg/ml): WKY: 302.76 ± 13.7684; SHR-C: 755.14 ± 33.34; SHR-B: 352.04 ± 22.50; *p* < 0.05 vs. WKY group; Table 1). However, BGP-15 treatment caused a marked reduction of the BNP level in hypertensive animals (*p* < 0.05, SHR-B vs. SHR-C).

#### 3.1.2. Effect of BGP-15 Administration on Mitochondrial Ultrastructure

Longitudinal sections of the myocardium were evaluated to assess the status of interfibrillar mitochondria (IFM) by electron microscopy. The mitochondria of SHR-C rats differ from the normal mitochondria of WKY rats (Figures 2(a)–2(c)), because they are morphologically more heterogeneous (*n* = 5 from each group, 3–5 block from each animal). In the nontreated hypertensive animals (SHR-C), mitochondria were loosely arranged between the contractile elements (Figures 3(a) and 3(b)). Moreover, in the SHR-C group, extensive disruption of mitochondrial cristae and enlarged intracristal spaces could be observed (Figure 3(c)). Their shape was often elongated, and the mitochondrial matrix was very light. The mitochondrial ultrastructure in the SHR-B group was similar to that of WKY rats (Figures 3(d) and 3(e)). In treated SHR animals (SHR-B), normal, large, and less elongated mitochondria with tightly packed cristae and electron-dense matrix were seen (Figure 3(f)). The area of IFM was assessed on electron micrographs (~500 mitochondria/group were measured; Figure 4(b)). We assessed relative frequencies of the measured mitochondrial areas in arbitrary intervals of 0.3 *μ*m^2^ (Figure 4(a)). In all the groups, less than 1% of mitochondrial areas were above the 1.81 *μ*m^2^ value. In the SHR-C group, 43.7% of the measured mitochondria belonged to the lowest area range (<0.3 *μ*m^2^). However, in the WKY group, the predominant area range of the measured mitochondria was between 0.3 and 0.6 *μ*m^2^. Due to BGP-15 treatment (SHR-B), the distribution of mitochondria was similar to that of the WKY group and the highest number of mitochondria (48%) belonged to the 0.3-0.6 *μ*m^2^ range (*p* < 0.05, SHR-B vs. SHR-C). Our results showed a profound decrease in the mean mitochondrial area of SHR-C group compared to the mitochondria of WKY animals (*p* < 0.05, SHR-C, vs. WKY). The values of BGP-15-treated SHRs differed from that of the SHR-C group (*p* < 0.05), and it was similar to the mitochondria of normotensive animals (WKY).

#### 3.1.3. Effect of BGP-15 Treatment on Mitochondrial Fusion Proteins in SHR Animals

Regarding the mitochondrial fusion proteins, we determined the levels of OPA1, MFN1, and MFN2 in the myocardium using Western blot analysis (Figure 5). We observed that the level of OPA1 was moderately decreased in the SHR-C group compared to the WKY group (*p* < 0.05, SHR-C vs. WKY). However, BGP-15 treatment caused a significant elevation of OPA1 level in the SHR-B group (*p* < 0.01 SHR-B vs. WKY, *p* < 0.05 SHR-B vs. SHR-C). Considering the amount of MFN1 protein level, there was a significant increase in hypertensive animals by the end of the study compared to the baseline levels (*p* < 0.05, SHR-C and SHR-B vs. SHR-Baseline); however, there was no difference between the SHR groups. The level of MFN2 protein was moderately lower in the SHR-C group than in the WKY group (*p* < 0.05), as observed in the case of OPA1. In the SHR-B group, this parameter increased significantly due to the treatment compared to the other groups (*p* < 0.01 SHR-B vs WKY, SHR-C).

#### 3.1.4. Effect of BGP-15 Administration on Mitochondrial Fission Proteins in SHR Animals

The levels of fission proteins Fis1 and DRP1 were determined in the myocardium in total and in fractionated Western blot samples (Figure 6). The level of Fis1 increased in the SHR-C group compared to the WKY group (*p* < 0.05, SHR-C vs. WKY). This elevation was, however, diminished significantly due to BGP-15 treatment (*p* < 0.05 SHR-B vs. SHR-C). In the case of the fission protein DRP1, the total level was significantly decreased due to BGP-15 treatment compared to other groups (*p* < 0.01 SHR-B vs. WKY, SHR-C). The phosphorylation level of DRP1 at the Ser616 and Ser637 residues was also measured. The phosphorylation of DRP1^Ser616^ and DRP1^Ser637^ was moderate in the WKY group. In the SHR-C group, however, phosphorylation of DRP1^Ser616^ was increased significantly (*p* < 0.01 vs. WKY and SHR-Baseline). BGP-15 treatment decreased DRP1^Ser616^ phosphorylation in SHR-B animals (*p* < 0.01 vs. SHR-C group). Regarding the phosphorylation level of DRP1^Ser637^, we observed a significant increase in the SHR-C group (*p* < 0.01 vs. WKY, SHR-Baseline). Moreover, BGP-15 treatment caused a further increase in the DRP1^Ser637^ phosphorylation in SHR-B animals (*p* < 0.01 SHR-B vs. SHR-C).

The intracellular distribution of DRP1 was also measured (Figure 7). We observed that the Drp1 accumulated in the mitochondrial fractions of SHR-C animals compared to normotensive animals (*p* < 0.01, SHR-C vs. WKY). BGP-15 treatment resulted in a significantly reduced translocation of Drp1 into the mitochondria (*p* < 0.01 vs. SHR-C), thereby preserving it in a higher concentration in the cytosolic fraction.

### 3.2. In Vitro Results

#### 3.2.1. Effect of BGP-15 Administration on Mitochondrial Morphology of NRCM Cells

To examine the changes of the mitochondrial network, we used the MitoTracker Red CMXRos staining method (Figure 8). BGP-15 per se had no effect on the complexity of the mitochondrial network. Filamentous mitochondrial network was observed in the Control group; H_2_O_2_ treatment, however, caused a marked injury to the mitochondrial network. As a result of the H_2_O_2_-induced fission processes, degradation of the mitochondrial network could be observed which led to mitochondrial fragmentation. BGP-15 treatment prevented the mitochondrial network from the oxidative stress-induced fragmentation and preserved the normal filamentous network of mitochondria.

#### 3.2.2. Effect of BGP-15 Treatment on Mitochondrial Fusion Proteins in NRCMs

We assessed the levels of OPA1, MFN1 and MFN2 proteins in total Western blot samples of NRCM cells (Figure 9). BGP-15 treatment per se had no effect in the nonstressed cells in comparison to the Control group. H_2_O_2_ treatment caused a slight decrease in the level of MFN1 and MFN2 proteins and a slight increase in the level of OPA1, but these changes were not significant. BGP-15 treatment caused a significant increase of OPA1, MFN1, and MFN2 proteins in H_2_O_2_ stressed cells compared to the H_2_O_2_-stressed group (*p* < 0.05 H_2_O_2_-BGP15 vs. H_2_O_2_).

#### 3.2.3. Effect of BGP-15 Administration on Mitochondrial Fission Proteins in NRCMs

We determined the levels of Fis1 and DRP1 in total and in fractionated Western blot samples in NRCM cells (Figure 10). No significant difference was found with BGP-15 treatment in nonstressed cells compared to the Control group. The level of Fis1 increased markedly in the H_2_O_2_ group compared to the Control group (*p* < 0.01, H_2_O_2_ vs. Control). Due to BGP-15 treatment, this change was blunted (*p* < 0.05, H_2_O_2_-BGP15 vs. H_2_O_2_ group). The case of the fission mediator DRP1 protein total level was a significant elevation in the H_2_O_2_ group due to oxidative stress (*p* < 0.05H_2_O_2_ vs. Control group). However, a control-like value could be seen in the treated group compared to the H_2_O_2_ group (*p* < 0.05 H_2_O_2_-BGP15 vs. H_2_O_2_ group). The phosphorylation of DRP1 on Ser616 and Ser637 residues was also evaluated. The phosphorylation of both DRP1 phospho-form was moderate in the Control group. Phosphorylation of DRP1^Ser616^ increased considerably in the H_2_O_2_ group (*p* < 0.05 H_2_O_2_ vs. Control group). However, BGP-15 treatment decreased DRP1^Ser616^ phosphorylation compared to nontreated stressed cells (*p* < 0.05 H_2_O_2_-BGP-15 vs. H_2_O_2_ group). Measuring the phosphorylation level of DRP1^Ser637^, a significant decrease could be observed in the H_2_O_2_ group compared to the Control group (*p* < 0.01 H_2_O_2_ vs. Control group). However, BGP-15 treatment enhanced remarkably the DRP1^Ser637^ phosphorylation (*p* < 0.01 H_2_O_2_-BGP15 vs. H_2_O_2_ group).

Finally, the intracellular distribution of fission mediator DRP1 protein was examined (Figure 11). A significantly higher portion of DRP1 could be found in the mitochondrial fraction of cells in the H_2_O_2_ group compared to the BGP-15-treated group. The translocation of DRP1 protein from the cytosol to the mitochondria was moderated as a result of the BGP-15 treatment and in this way resulted in higher levels of DRP1 in the cytosolic fraction and lower concentration in the mitochondrial fraction (*p* < 0.01 vs. H_2_O_2_ group).

#### 3.2.4. Effect of BGP-15 Treatment on the Regulatory Factors of Mitochondrial Biogenesis in NRCMs

We determined the levels of PGC-1*α*, CREB and VDAC in the total Western blot samples of NRCMs. BGP-15 treatment had no effect on these factors in nonstressed cells compared to the Control group. The PGC-1*α* level was increased in the H_2_O_2_ group compared to the Control group (*p* < 0.01 vs. Control; Figure 12). However, this elevation was much more marked in the treated group (*p* < 0.01 H_2_O_2_-BGP15 vs. Control and H_2_O_2_ groups). The phosphorylation level of CREB^Ser133^ was low in the Control group. However, a significant increase was seen in the phosphorylation level of CREB^Ser133^ in the H_2_O_2_ group (*p* < 0.01 H_2_O_2_ vs. Control) (Figure 12). BGP-15 treatment increased further the phosphorylation level of CREB^Ser133^ (*p* < 0.01, H_2_O_2_-BGP15 vs. H_2_O_2_ group). The level of VDAC was slightly decreased in the H_2_O_2_ group compared to the Control group (*p* < 0.05 H_2_O_2_ vs. Control). The level of the VDAC, however, was significantly elevated in the BGP-15 treated group (*p* < 0.01 H_2_O_2_-BGP-15 vs. H_2_O_2_ group).

Moreover, we investigated mitochondrial DNA content compared to the nuclear DNA. The relative mitochondrial DNA content was determined by “real-time” PCR, using COX1 and COX3 primers, normalized to a nuclear-encoded *β*-actin gene. We found that BGP-15 treatment increased the relative expression levels of COXI and COXIII genes compared to the H_2_O_2_ group (*p* < 0.05 H_2_O_2_-BGP-15 vs. H_2_O_2_ group; Figure 13).

Furthermore, we also performed a well-accepted method for studying mitochondrial biogenesis by measuring the activity of citrate synthase (Figure 13). Citrate synthase activity was reduced in hydrogen-peroxide stressed group compared to the control group (*p* < 0.01 H_2_O_2_ vs. Control). The citrate synthase activity was increased significantly due to the treatment (*p* < 0.01 H_2_O_2_-BGP-15 vs. H_2_O_2_ group; Figure 13).

Finally, we measured the level of NDUFs1 subunit of NADH-ubiquinone oxidoreductase and UQCRC1 subunit of Ubiquinol Cytochrome c Reductase proteins in order to support our finding regarding the effect of BGP-15 on mitochondrial biogenesis. The expression level of NDUFs1 was significantly decreased in the H2O2 group (*p* < 0.01 H_2_O_2_ vs. Control; Figure 14). A similar observation was made in the case of UQCRC1 (*p* < 0.05 H_2_O_2_ vs. Control). However, BGP-15 treatment not only protected against the decrease but also significantly increased the amount of NDUFs1 and UQCRC1 proteins (*p* < 0.01 H_2_O_2_-BGP-15 vs. H_2_O_2_ group).

#### 3.2.5. Effect of BGP-15 Administration on Mitochondrial Genome Integrity

Real-time detection of long-range polymerase chain reaction (LRPCR) was used to examine the impact of H_2_O_2_-induced oxidative injury on mtDNA (Figure 15). No significant difference was found with BGP-15 treatment alone compared to the Control group. H_2_O_2_ induced a significant damage of the mtDNA (*p* < 0.05, H_2_O_2_ vs. Control); the amplification rate of the entire mitochondrial genome was markedly diminished. This unfavourable damage was significantly reduced by BGP-15 treatment (*p* < 0.01, H_2_O_2_-BGP15 vs. H_2_O_2_).

#### 3.2.6. Effect of BGP-15 on Mitochondrial Membrane Potential (*ΔΨ*) in NRCM Cells

We examined the effect of BGP-15 on mitochondrial membrane potential using JC-1, a cell-permeable voltage-sensitive fluorescent mitochondrial dye (Figure 16). JC-1 emits red fluorescence if the mitochondrial membrane potential is high (aggregated dye), while depolarized mitochondria emit green fluorescence (monomer dye). In the control cells, fluorescence microscopy showed strong red fluorescence and weak green fluorescence, which indicates a high *ΔΨ*m in mitochondria (Figure 16(a)). BGP-15 per se had no effect on mitochondrial membrane potential. The addition of H_2_O_2_ to cells facilitates the depolarization of mitochondria, resulting in weaker red fluorescence and stronger green fluorescence (*p* < 0.01 H_2_O_2_ vs. Control; Figure 16(b)). If BGP-15 was also administered in peroxide-stressed NRCM cells, red fluorescence increased and green fluorescence decreased compared to the H_2_O_2_-treated cells (*p* < 0.01, H_2_O_2_-BGP15 vs. H_2_O_2_) (Figure 16(b)). Therefore, the quantitative assessment revealed that BGP-15 treatment reduced the H_2_O_2_-induced depolarization of the mitochondrial membrane; the *ΔΨ*m was similar to that of the Control cells.

#### 3.2.7. Effect of BGP-15 on Mitochondrial Oxygen Consumption and Energy Metabolism in NRCM Cells

To determine the mitochondrial energy metabolism and respiratory function, we used the Agilent Seahorse XFp Analyzer system and the Agilent Seahorse XFp Cell Mito Stress Test (Figure 17). BGP-15 itself had no effect on the rate of mitochondrial respiration. The oxygen consumption rate of NRMC cells was decreased in the presence of H_2_O_2_ to cells compared to Control cells (Figure 17(a)). H_2_O_2_ treatment decreased the basal respiration although this difference was not significant (Figure 17(b)). However, the maximal respiration, the spare respiratory capacity, and the ATP production were markedly decreased as a result of H_2_O_2_-induced oxidative damage compared to the Control group (*p* < 0.05, H_2_O_2_ vs. Control) (Figures 17(c)–17(e)). In the presence of both H_2_O_2_ and BGP-15, the maximal respiration, spare respiratory capacity, and the ATP production were significantly higher compared to the H_2_O_2_ group (*p* < 0.05, H_2_O_2_–BGP15 vs. H_2_O_2_).

## 4. Discussion

We aimed to study the effect of BGP-15 on various processes of mitochondrial quality control in a hypertension-induced heart failure model and in vitro using hydrogen peroxide-induced oxidative stress. The major findings of this study are that BGP-15, besides its promoting effect on mitochondrial fusion, also inhibits factors playing part in the mitochondrial fission and enhances their de novo biogenesis under stress situations. As a result of these effects, BGP-15 preserves mitochondrial structure and energy production during hydrogen peroxide-induced oxidative stress as well as in an in vivo heart failure model.

In our recent work, spontaneously hypertensive rats (SHR) were used, which is a widely used model in experimental cardiology for the examination of hypertension-induced cardiovascular remodelling and heart failure [26–28]. 15-month-old SHRs showed already severe left ventricular hypertrophy with mild signs of heart failure. BGP-15 has a positive effect on remodelling processes and cardiac function [29]. In our work, BGP-15 treatment decreased slightly the severity of cardiac hypertrophy, which was proved by gravimetric parameters (weight of ventricles/body weight, weight of ventricles/tibia length) and decreased the severity of heart failure characterized by BNP level (Table 1). In the background of these favourable changes, the mitochondrial structural and functional alterations were assumed.

Mitochondria are dynamic organelles constantly undergoing fusion and fission processes. Hypertension-induced heart failure is characterized by the fragmentation of mitochondria and by compromised energy production leading to decreased contractile force of myofilaments [30, 31]. In our work, mitochondria were structurally damaged in nontreated hypertensive animals (SHR-C). They were loosely arranged between the contractile elements (Figures 3(a)–3(c)). The average size of mitochondria was markedly reduced in the SHR-C group; approximately 40% of mitochondria were smaller than 0.3 *μ*m2 as a result of heart failure-induced mitochondrial fragmentation (Figures 4(a)–4(c)). Ultrastructurally, extensive disruption of mitochondrial cristae and enlarged intracristal spaces was observed. However, BGP-15 treatment resulted in structurally markedly healthier mitochondria that were similar to that of normotensive animals. Mitochondria in the SHR-B group were tightly packed between the myofibrils. Most of mitochondria belonged to the normal size range (0.3-0.6 *μ*m2), which can be—at least partially—the consequence of increased mitochondrial biogenesis. On the ultrastructural level, large mitochondria with tightly packed cristae and electron-dense matrix were seen in the treated group (Figures 3(d)–3(f)).

Oxidative stress induces an imbalance in processes of mitochondrial dynamics, potentially leading to cell death. Proper mitochondrial functions regulated by the quality control processes are fundamental for cardiac work. The deterioration of mitochondrial quality control greatly contributes to the hypertension-induced cardiac remodelling and its progression to heart failure [4, 7, 8]. In our recent study, the expression level of proteins promoting the mitochondrial fusion, particularly OPA1 and MFN2, was increased significantly in the BGP-15-treated animals compared to the SHR-C group (Figure 5). Our results are in accordance with the results of Szabo et al., who published earlier that BGP-15 has promoted mitochondrial fusion in both in vitro and in vivo [18].

Regarding mitochondrial fission, a marked decrease could be seen in the expression levels of DRP1 and Fis1 in hypertensive animals due to BGP-15 treatment (Figure 6). DRP1 is regulated by several posttranslational modifications [32–34]. DRP1^Ser637^ phosphorylation suppresses its translocation to mitochondria and thus inhibits its activity, while DRP1^Ser616^ phosphorylation promotes DRP1 translocation and therefore the mitochondrial fission. BGP-15 treatment increased markedly the DRP1^Ser637^ phosphorylation and decreased the DRP1^Ser616^ phosphorylation in SHR-B animals compared to nontreated hypertensive animals (Figure 6). The subcellular distribution of DRP1 showed changes consistent with the phosphorylation pattern of DRP1. In nontreated hypertensive animals (SHR-C), a high portion of DRP1 could be observed in the mitochondrial fraction (Figure 7). BGP-15 treatment resulted in a significantly reduced translocation to mitochondria of DRP1, retaining it in the cytosolic fraction. This can be a consequence of increased DRP1^Ser637^ phosphorylation in SHR-B animals. Altogether, BGP-15 prevented mitochondria against hypertension-induced fragmentation.

In our in vitro experiments, hydrogen-peroxide was used to induce oxidative injury of NRCM cells. Degradation of the filamentous mitochondrial network by mitochondrial fragmentation could be observed in H_2_O_2_-stressed NRCM cells. BGP-15 treatment prevented the mitochondrial network from the oxidative stress-induced fragmentation and preserved mitochondria predominantly in the filamentous state.

Similar changes were seen in the case of fusion and fission processes in NRCM cell culture compared to in vivo model. BGP-15 treatment increased the expression level of fusion proteins (OPA1, MFN1, and MFN2), and thus, it can promote mitochondrial fusion during oxidative stress (Figure 9). On the other hand, the level of fission mediators (DRP1 and Fis1) was decreased due to BGP-15 treatment (Figure 10). BGP-15 also moderated the mitochondrial translocation of DRP1 protein from the cytosol as a result of enhanced DRP1^Ser637^ phosphorylation and decreased phosphorylation of DRP1^Ser616^ (Figure 11). Therefore, BGP-15 treatment has beneficial effects on mitochondrial dynamics by promoting the fusion and blocking the fission processes.

Several studies have demonstrated that mitochondrial biogenesis is compromised in cardiac remodelling and heart failure [35–37]. PGC-1-*α* is the key regulator of biogenesis, which in turn is regulated by CREB [38–40]. We found that the expression level of PCG-1*α* increased significantly due to BGP-15 treatment (Figure 12). Moreover, BGP-15 treatment further enhanced the phosphorylation of CREB compared to H_2_O_2_ group, too (Figure 12). CREB increased the expression level of PGC-1*α* and therefore can enhance mitochondrial biogenesis. VDAC is located in the outer mitochondrial membrane and can be used for mitochondrial loading protein. We found that VDAC was significantly elevated in BGP-15-treated cells that can support our previous results regarding enhanced biogenesis.

Moreover, we examined the level of NDUFs1 subunit of NADH-ubiquinone oxidoreductase and UQCRC1 subunit of Ubiquinol Cytochrome c Reductase proteins. These proteins are part of the mitochondrial electron transport chain (ETC Complex I and III), and in this way, they are essentially important in the maintaining of proper mitochondrial function [41, 42]. The amount of ETC Complex I and Complex III proteins levels was increased significantly due to BGP-15 treatment, which is consistent with our previous results (Figure 14).

In order to support our finding more adequately regarding the effect of BGP-15 on mitochondrial biogenesis, the relative DNA content of ETC Complex IV was determined. We found that BGP-15 treatment increased the relative expression levels of both tested genes (COXI and COXIII; Figure 13). Since both genes are encoded by mitochondrial DNA, this suggests that mitochondrial DNA content was increased in NRCMs cells treated with BGP-15.

Moreover, we also performed a well-accepted and frequently used method for studying mitochondrial biogenesis by measuring the activity of citrate synthase (CS) [43–45]. Citrate synthase is localized within the mitochondrial matrix, and it catalyses the synthesis of citrate from oxaloacetate in the Krebs tricarboxylic acid cycle [44]. Maximal activity of citrate synthase indicates the mitochondrial content of heart muscle. Citrate synthase activity was reduced in hydrogen-peroxide stressed group compared to control group. The citrate synthase activity was increased significantly due to the treatment (Figure 13). Summarizing these results, we can conclude that mitochondrial biogenesis was increased under oxidative stress in treated NRCMs cells as a result of BGP-15 treatment, and in this way, it was able to enhance the proper mitochondrial function.

Oxidative stress can damage the mtDNA, which is extremely sensitive to it [46, 47]. In our recent work, PCR results showed extensive damage of mtDNA caused by hydrogen peroxide. Thus, the amplification of the entire mitochondrial genome was restrained. BGP-15 treatment, however, preserved mitochondrial genome integrity markedly decreasing the breakage of mtDNA (Figure 15). The protection of mtDNA is extremely important, because the mitochondrial respiratory chain (ETC) complexes are encoded on mtDNA [48, 49]. Complex I-III are critical for ROS production by the respiratory chain [50]. It can generate significant amounts of ROS under several conditions including hypoxia, mitochondrial hyperpolarization, and inhibition of respiratory complexes. BGP-15 is able to reduce the mitochondrial ROS production at complex I [18, 24]. Along these lines, BGP-15 can protect against ROS induced mitochondrial DNA damage and maintain the appropriate mitochondrial function.

The preservation of mitochondrial membrane potential is also important to maintain the metabolic capacity of mitochondria. Well-functioning mitochondrial oxidative phosphorylation and ATP production are essential for the proper function of cardiomyocytes [51, 52]. BGP-15 is able to prevent oxidative stress-induced mitochondrial membrane potential loss and therefore improved mitochondrial function (Figure 16). We observed that oxidative stress leads to mitochondrial respiration damage (Figure 17). However, BGP-15 treatment preserved the mitochondrial function characterized by ATP production and spare respiratory capacity thereby ensuring the ability of cells to respond to increased energy demand under stress scenario.

BGP-15 also supports the maintenance of mitochondrial function partially via the preservation of the mitochondrial structure.

Our study is the first to demonstrate that BGP-15 preserved the mitochondrial ultrastructure by increased mitochondrial fusion and decreased fission processes as well as positively affected the translocation processes in chronic hypertension-induced heart failure animal model. Furthermore, we can make a similar observation in the case of primer rat cardiomyocytes cell culture experiment during hydrogen-peroxide induced oxidative stress. Comparable changes were seen in the case of fusion and fission processes in NRCM cell culture compared to in vivo model. Moreover, BGP-15 treatment preserved the mitochondrial membrane potential and improved the mitochondrial function. BGP-15 protected the integrity of the mitochondrial genome and enhanced the de novo biogenesis of mitochondria during hydrogen peroxide-induced oxidative stress. Nevertheless, the exact molecular mechanism of the effects is still unknown, but there are clear evidences regarding the specific mechanism of how BGP-15 acts at important integrator points of signal transduction in certain pathological processes. In order to elucidate the potential underlying molecular mechanisms, further targeted studies should be performed in the future.

Our results reveal that pharmacological modulation of the mitochondrial dynamics under cellular stress could be a novel therapeutic approach in various cardiac diseases characterized by oxidative stress-induced mitochondrial damage.

## Figures and Tables

**Figure 1:** Chemical structure of BGP-15 (O-[3-piperidino-2-hydroxy-1-propyl]-nicotinic acid amidoxime dihydrochloride) [24].

**Figure 2:** Ultrastructural analysis of interfibrillar mitochondria in the myocardium of WKY animals. Representative electron micrographs of interfibrillar mitochondria in the myocardium of (a, b) WKY animals ((a) magnification: 15 k, scale bar: 0.2 *μ*m; (b) magnification: 20 k, scale bar: 0.2 *μ*m). Ultrastructure of interfibrillar mitochondria in the myocardium of (c) WKY animals (magnification: 40 k, scale bar: 0.1 *μ*m (*n* = 4 from each group, 3–5 blocks from each animal). WKY: age-matched normotensive Wistar-Kyoto rats.

**Figure 3:** Ultrastructural analysis of interfibrillar mitochondria in the myocardium of SHR animals. Representative electron micrographs of interfibrillar mitochondria in the myocardium of (a, b) SHR-C and (d, e) SHR-B animals (magnification: 10 k, scale bar: 1 *μ*m). Ultrastructure of interfibrillar mitochondria in the myocardium of (c) SHR-C and (f) SHR-B animals (magnification: 25 k, scale bar: 0.5 *μ*m). SHR-C: nontreated spontaneously hypertensive rats; SHR-B: spontaneously hypertensive rats receiving BGP-15 for 18 weeks (*n* = 4 from each group, 3–5 blocks from each animal).

**Figure 4:** Heart failure-induced fragmentation of interfibrillar mitochondria in the myocardium. (a) Relative frequencies of measured mitochondrial areas in each arbitrary area interval. (b) Means of area values in given groups (~500 mitochondria/group). WKY: age-matched normotensive Wistar-Kyoto rats; SHR-C: nontreated spontaneously hypertensive rats; SHR-B: spontaneously hypertensive rats receiving BGP-15 for 18 weeks. Data are expressed as mean ± SEM. ^∗^*p* < 0.05 vs. WKY, ^§^*p* < 0.05 vs. SHR-C.

**Figure 5:** Effect of BGP-15 treatment on mitochondrial fusion proteins in a hypertension-induced heart failure model. Western blot analysis of OPA1, MFN1, and MFN2 proteins as well as densitometric evaluations is shown. GAPDH was used as a loading control. WKY: age-matched normotensive Wistar-Kyoto rats; SHR-Baseline: 15-month-old spontaneously hypertensive rats; SHR-C: 19-month-old nontreated spontaneously hypertensive rats; SHR-B: 19-month-old spontaneously hypertensive rats receiving BGP-15 for 18 weeks (*n* = 4). Values are mean ± SEM. ^∗^*p* < 0.05 vs. WKY, ^∗∗^*p* < 0.01 vs. WKY, ^##^*p* < 0.01 vs. SHR-Baseline, ^§§^*p* < 0.01 vs SHR-C.

**Figure 6:** Effect of BGP-15 treatment on mitochondrial fission proteins in a hypertension induced-heart failure model. Western blot analysis of Fis1 and DRP1 proteins, as well as densitometric evaluation, is shown. GAPDH was used as a loading control. WKY: age-matched normotensive Wistar-Kyoto rats; SHR-Baseline: 15-month-old spontaneously hypertensive rats; SHR-C: 19-month-old nontreated spontaneously hypertensive rats; SHR-B: 19-month-old spontaneously hypertensive rats receiving BGP-15 for 18 weeks (*n* = 4). Values are mean ± SEM. ^∗^*p* < 0.05 vs. WKY, ^∗∗^*p* < 0.01 vs. WKY, ^##^*p* < 0.01 vs. SHR-Baseline, ^§^*p* < 0.05 vs. SHR-C, ^§§^*p* < 0.01 vs. SHR-C.

**Figure 7:** Effect of BGP-15 treatment on DRP1 protein intracellular distribution in a hypertension-induced heart failure model. Western blot analysis regarding the intracellular distribution of DRP1 protein and densitometric evaluation are also shown. GAPDH and PDC were used as a loading control. WKY: age-matched normotensive Wistar-Kyoto rats; SHR-Baseline: 15-month-old spontaneously hypertensive rats; SHR-C: 19-month-old nontreated spontaneously hypertensive rats; SHR-B: 19-month-old spontaneously hypertensive rats receiving BGP-15 for 18 weeks (*n* = 4). Values are mean ± SEM. ^∗∗^*p* < 0.01 vs. WKY, ^§§^*p* < 0.01 vs SHR-C.

**Figure 8:** Effect of BGP-15 administration on the morphology of mitochondrial network in NRCM cells. For methodical details, see chapter “Materials and Methods.” BGP-15 treatment prevented the mitochondrial network from the oxidative stress-induced fragmentation and preserved mitochondria predominantly in the normal filamentous state. The inserts show the filamentous and fragmented states, showing that BGP-15 protected the mitochondrial network. Control group: cells without any treatment; BGP-15 group: cells with only 50 *μ*M BGP-15 for 0.5 hours; H_2_O_2_ group: cells with 150 *μ*M H_2_O_2_ for 0.5 hours; H_2_O_2_+BGP-15 group: cells with 150 *μ*M H_2_O_2_ and 50 *μ*M BGP-15 for 0.5 hours.

**Figure 9:** Effect of BGP-15 treatment on mitochondrial fusion proteins in NRCM cells. Western blot analysis of OPA1, MFN1, and MFN2 as well as densitometric evaluation is shown. GAPDH was used as a loading control. Control group: cells without any treatment; BGP-15 group: cells with only 50 *μ*M BGP-15 for 0.5 hours; H_2_O_2_ group: cells with 150 *μ*M H_2_O_2_ for 0.5 hours; H_2_O_2_+BGP-15 group: cells with 150 *μ*M H_2_O_2_ and 50 *μ*M BGP-15 for 0.5 hours. Values are mean ± SEM (*n* = 4). ^∗^*p* < 0.05 vs. Control, ^§^*p* < 0.05 vs. H_2_O_2_ group.

**Figure 10:** Effect of BGP-15 treatment on mitochondrial fission proteins in NRCM cells. Western blot analysis of Fis1 and DRP1 proteins, as well as densitometric evaluation, is shown. GAPDH was used as a loading control. Control group: cells without any treatment, BGP-15 group: cells with only 50 *μ*M BGP-15 for 0.5 hours; H_2_O_2_ group: cells with 150 *μ*M H_2_O_2_ for 0.5 hours; H_2_O_2_+BGP-15 group: cells with 150 *μ*M H_2_O_2_ and 50 *μ*M BGP-15 for 0.5 hours. Values are mean ± SEM (*n* = 4). ^∗^*p* < 0.05 vs. Control, ^∗∗^*p* < 0.01 vs. Control, ^§^*p* < 0.05 vs. H_2_O_2_ group, ^§§^*p* < 0.01 vs. H_2_O_2_ group.

**Figure 11:** Effect of BGP-15 treatment on intracellular distribution of DRP1 protein in stressed NRCM cells. Western blot analysis of DRP1 protein regarding its intracellular disruption, as well as densitometric evaluation, is shown. GAPDH and PDC were used as a loading control. Control group: cells without any treatment; BGP-15 group: cells with only 50 *μ*M BGP-15 for 0.5 hours; H_2_O_2_ group: cells with 150 *μ*M H_2_O_2_ for 0.5 hours; H_2_O_2_+BGP-15 group: cells with 150 *μ*M H_2_O_2_ and 50 *μ*M BGP-15 for 0.5 hours. Values are mean ± SEM (*n* = 4). ^∗∗^*p* < 0.01 vs. Control, ^§§^*p* < 0.01 vs. H_2_O_2_ group.

**Figure 12:** Effect of BGP-15 treatment on the regulation of mitochondrial biogenesis in NRCM cells. Western blot analysis of PGC-1-*α*, CREB, and VDAC proteins as well as densitometric evaluation is shown. GAPDH was used as a loading control. Control group: cells without any treatment; BGP-15 group: cells with only 50 *μ*M BGP-15 for 0.5 hours; H_2_O_2_ group: cells with 150 *μ*M H_2_O_2_ for 0.5 hours; H_2_O_2_+BGP-15 group: cells with 150 *μ*M H_2_O_2_ and 50 *μ*M BGP-15 for 0.5 hours. Values are mean ± SEM (*n* = 4). ^∗^*p* < 0.05 vs. Control, ^∗∗^*p* < 0.01 vs. Control, ^§§^*p* < 0.01 vs H_2_O_2_ group.

**Figure 13:** Effect of BGP-15 treatment on the relative DNA content and citrate synthase activity. Relative expression level of electron transport chain complex IV genes (COX1 and COX3 are presented. Comparison of citrate synthase activity in NRCM cells. Control group: cells without any treatment; BGP-15 group: cells with only 50 *μ*M BGP-15 for 0.5 hours, H_2_O_2_ group: cells with 150 *μ*M H2O2 for 0.5 hours, H2O2+BGP-15 group: cells with 150 *μ*M H_2_O_2_ and 50 *μ*M BGP-15 for 0.5 hours. Values are mean ± SEM (*n* = 4). ^∗∗^*p* < 0.01 vs. Control, ^§§^*p* < 0.01 vs. H_2_O_2_ group.

**Figure 14:** Effect of BGP-15 treatment on the electron transport chain complex I and III proteins in NRCMs. Western blot analysis of UQCRC1 and NDUFs1 proteins as well as densitometric evaluation is shown. GAPDH was used as a loading control. Control group: cells without any treatment; BGP-15 group: cells with only 50 *μ*M BGP-15 for 0.5 hours; H_2_O_2_ group: cells with 150 *μ*M H_2_O_2_ for 0.5 hours; H_2_O_2_+BGP-15 group: cells with 150 *μ*M H_2_O_2_ and 50 *μ*M BGP-15 for 0.5 hours. Values are mean ± SEM (*n* = 4). ^∗^*p* < 0.05 vs. Control, ^∗∗^*p* < 0.01 vs. Control, ^§§^*p* < 0.01 vs H_2_O_2_ group.

**Figure 15:** Effect of BGP-15 treatment on oxidative stress-induced mitochondrial DNA damage. Total DNA was isolated for LRPCR and SRPCR analysis. mtDNA damage was calculated using the *Δ*2^Ct^ method. Control group: cells without any treatment; BGP-15 group: cells with only 50 *μ*M BGP-15 for 0.5 hours; H_2_O_2_ group: cells with 150 *μ*M H_2_O_2_ for 0.5 hours; H_2_O_2_+BGP-15 group: cells with 150 *μ*M H_2_O_2_ and 50 *μ*M BGP-15 for 0.5 hours. Values are mean ± SEM (*n* = 4). ^∗^*p* < 0.05 vs. Control, ^§§^*p* < 0.01 vs H_2_O_2_ group.

**Figure 16:** Effect of BGP-15 on the mitochondrial membrane potential in NRCMs, as determined by JC-1. (a) Effect of BGP-15 on H_2_O_2_-induced mitochondrial membrane depolarization in NRCM cells. Cells were exposed to 150 *μ*m H_2_O_2_ in the absence or presence of 50 *μ*m BGP-15 for 0.5 hours, after that stained with 100 ng/ml of JC-1. The dye was loaded, and after a 15-minute-long incubation, fluorescent microscopic images were taken using both the red and green channels. Representative merged images are presented. (b) Quantitative analysis of mitochondrial depolarization induced by H_2_O_2_ (150 *μ*M) and its reduction by BGP-15 (50 *μ*M) in NRCM cells. Control group: cells without any treatment; BGP-15 group: cells with only 50 *μ*M BGP-15 for 0.5 hours; H_2_O_2_ group: cells with 150 *μ*M H_2_O_2_ for 0.5 hours; H_2_O_2_+BGP-15 group: cells with 150 *μ*M H_2_O_2_ and 50 *μ*M BGP-15 for 0.5 hours. Data are presented as the mean ± SEM. ^∗∗^*p* < 0.01 vs. Control cells; ^§§^*p* < 0.01 vs H_2_O_2_-treated cells.

**Figure 17:** Effect of BGP-15 on mitochondrial oxygen consumption and energy metabolism in NRCM cells, as determined by Agilent Seahorse Xfp. Mitochondrial energy metabolism was measured using a Seahorse XFp analyzer. During testing, H9c2 cells were treated with 10 *μ*M oligomycin, 10 *μ*M FCCP, and 5 *μ*M rotenone/antimycin A. Data were automatically calculated according to the Agilent Seahorse XF Cell Mito Stress Test Report Generator. (a) Oxygen consumption rate (OCR). (b) Basal respiration. (c) ATP production. (d) Maximal respiration. (e) Spare respiratory capacity. Control group: cells without any treatment; BGP-15 group: cells with only 50 *μ*M BGP-15 for 0.5 hours; H_2_O_2_ group: cells with 150 *μ*M H_2_O_2_ for 0.5 hours; H_2_O_2_+BGP-15 group: cells with 150 *μ*M H_2_O_2_ and 50 *μ*M BGP-15 for 0.5 hours. Values are mean ± SEM (*n* = 4). ^∗^*p* < 0.05 vs. Control, ^§^*p* < 0.05 vs. H_2_O_2_ group.

**Table 1:** Effect of BGP-15 administration on gravimetric parameters and on BNP level of SHR animals.

	WKY	SHR-C	SHR-B
BW^START^ (g)	391.51 ± 8.64	340.66 ± 6.74^∗^	347.4 ± 10.38^∗^
BW^END^ (g)	403.22 ± 10.35	352.13 ± 6.86^∗^	365.29 ± 6.82^∗^
HW^END^ (g)	1.11 ± 0.03	1.41 ± 0.03^∗∗^	1.28 ± 0.02^∗∗^^,#^
VW^END^ (g)	0.98 ± 0.03	1.27 ± 0.02^∗^	1.12 ± 0.02^∗^
VW/BW^END^ (mg/g)	2.43 ± 0.07	3.60 ± 0.04^∗^	3.07 ± 0.09^∗^^,#^
VW/TL^END^ (mg/mm)	21.43 ± 0.71	29.14 ± 0.39^∗^	24.81 ± 0.53^∗^^,#^
p-BNP (pg/ml)	302.76 ± 13.77	755.15 ± 33.34^∗^	352.05 ± 22.50^#^

BW^START^: body weight at the beginning of the treatment; BW^END^: body weight at the end of the treatment; HW^END^: heart weight at the end of the treatment; VW^END^: ventricles weight at the end of the treatment; TL^END^: length of right tibia at the end of the treatment; p-BNP: plasma brain-type natriuretic peptide. Values are means + SEM. WKY: age-matched normotensive Wistar-Kyoto rats, *n* = 8, SHR-C: nontreated spontaneously hypertensive rats, *n* = 8, SHR-B: spontaneously hypertensive rats receiving BGP-15 for 18 weeks, *n* = 8. ^∗^*p* < 0.05 vs. WKY, ^∗∗^*p* < 0.01 vs. WKY, ^#^*p* < 0.05 vs. SHR-C.

## Data Availability

The authors confirm that all data is fully available without restriction. All relevant data is described within the paper.
